The article "High‐powered 675‐nm laser: Safety and efficacy in clinical evaluation and in vitro evidence for different skin disorders" was retracted in 2026. Reasons: compromised peer review; unreliable results or conclusions; lack of ethics approval or compliance.

# High‐powered 675‐nm laser: Safety and efficacy in clinical evaluation and in vitro evidence for different skin disorders

**DOI:** 10.1111/srt.70019

**Published:** 2024-08-29

**Authors:** Massimo D. F. Vitale, Francesca Madeddu, Irene Fusco, Laura Pieri, Paolo Bonan, Tiziano Zingoni, Giada Magni, Francesca Rossi

**Affiliations:** ^1^ Polyclinic of San Domenico Private Practice Bologna Italy; ^2^ El.En. Group Calenzano Italy; ^3^ Laser Cutaneous Cosmetic and Plastic Surgery Unit Villa Donatello Clinic Florence Italy; ^4^ Cnr – Istituto di Fisica Applicata “Nello Carrara” Via Madonna del Piano Sesto Fiorentino Italy

**Keywords:** acne scars, clinical skin rejuvenation management, high‐powered 675‐nm laser, pigmented lesions, in vitro experiments, confocal microscopy

## Abstract

**Background:**

Laser technology is a viable therapeutic option for treating a number of skin pathologic conditions, including pigmented lesions, vascular lesions and acne scars.

**Aim:**

In this work, through in vitro and clinical investigations we test the efficacy, the safety and the speed of treatment of high‐powered laser system emitting a 675‐nm in the management of various skin condition.

**Materials and methods:**

In vitro experiments were performed irradiating adult human dermal fibroblasts cells (HDFa) with 675‐nm laser for 24, 48 and 72 h with different fluences and Ki‐67^+^ cells were counted. The confocal microscopy images of control and treated samples were acquired. Clinical skin rejuvenation/diseases treatments with 675 nm laser device were performed with different laser parameters in 11 patients with pigmented lesions, 5 patients with acne scars and 23 patients for skin rejuvenation. Data were evaluated with the validated global score using 5‐point scales (GAIS) and patient's satisfaction scale.

**Results:**

The application of the high‐power 675 nm laser has proven effective in stimulating cell proliferation in in vitro experiments and it led to good results for all skin pathologies. GAIS showed values between 3 and 4 points for all treated pathologies, all scores between ‘75%‐good improvements’ and ‘100%‐excellent improvements’. The treatment time was reduced by 50% compared to the old parameters setting, resulting in a faster and good patient's satisfying technique. No serious adverse effects were recorded. Conclusion: the preclinical and clinical data confirm the efficacy and safety of this high‐powered 675 nm laser for several skin condition.

## 1 INTRODUCTION

Nowadays, several skin pathologic disorders such as acne scars, vascular lesions and pigmented lesions, can be treated with laser technology as a valid therapeutic alternative to conventional treatments.^1^ Topical formulations of traditional agents like hydroquinone, kojic acid, and glycolic acid are the first line of treatment for hyperpigmentation. These are followed by oral formulations of therapeutic agents including tranexamic acid, melatonin, and cysteamine hydrochloride. These treatments, however, have significant drawbacks, including the potential for erythema, skin peeling, and dryness, and they take a long time to produce noticeable results.^2^ Pathological scars can currently be treated using a variety of techniques, such as radiation therapy, medication therapy, surgery, and biological therapy. However, major obstacles still remain for these treatments, including a high risk of recurrence, significant side effects, and poor efficacy. Thus, there is an urgent requirement to find safer and more effective treatments.^3^

The article "High‐powered 675‐nm laser: Safety and efficacy in clinical evaluation and in vitro evidence for different skin disorders" was retracted in 2026. Reasons: compromised peer review; unreliable results or conclusions; lack of ethics approval or compliance.

Laser sources have been employed for numerous skin conditions during the past 50 years, and most dermatological specialties have seen an increase in their utilization. Laser technology allows physicians to treat a wide range of skin disorders, including inflammatory and neoplastic ones.^1^

Currently, a class of laser device known as non‐ablative lasers has been proposed, specifically in the fields of dermatology and aesthetic medicine. Its goal is to transfer energy to produce a photobiological impact rather than to destroy tissues. Using a technique known as ‘selective photo‐thermolysis’, these lasers use a specific wavelength absorbed differently by the various components of the skin, such as water, haemoglobin, and melanin, and producing a variety of biological effects. As a result, the energy of the absorbed photons is transferred to the irradiated tissue, leading to different biological effects at different scales, according to the applied dose.^4^, ^5^, ^6^ Among non‐ablative lasers, the 675‐nm device proved its efficacy in preclinical research.^7^, ^8^ In particular, on cultured fibroblast isolated from adult human derma, we demonstrated that the application of 390 J/cm^2^ stimulates the synthesis of type III collagen. At the same time, no cytotoxic effects were detected, as cell proliferation and viability remained unaffected in treated samples compared to non‐irradiated ones.

Given the fundamental role that fibroblasts play in the synthesis and deposition of collagen in the dermis,^9^ we have used another marker for the study of the effects of radiation emitted at 675 nm on the proliferation of these cells. Here, we used the Ki‐67 marker, known to be exploited in the detection of cell proliferation of pathological cells, but also in primary cultures and cell lines under physiological conditions.^10^, ^11^ Ki‐67 was originally identified in 1983 in L428 cells, a cell line of Hodgkin lymphoma in a laboratory in Kiel (Germany), in the sixty‐seventh well of a 96‐multiwell.^11^ The use of specific monoclonal antibodies allowed to characterize the expression of this protein at nuclear level only in proliferating cells, while it is absent in resting cells.^12^ In addition, the expression of Ki‐67 varies spatially within the cell nucleus during the different phases of the cell cycle.^13^ For this reason, Ki‐67 has immediately become a widely used diagnostic tool in the clinical field.^11^

The article "High‐powered 675‐nm laser: Safety and efficacy in clinical evaluation and in vitro evidence for different skin disorders" was retracted in 2026. Reasons: compromised peer review; unreliable results or conclusions; lack of ethics approval or compliance.

Furthermore, the 675‐nm laser device was tested in prospective observational clinical studies, applied in the management of facial rejuvenation,^14^ and in the treatment of acne vulgaris scars,^15^ additionally in dark‐skinned phototypes,^16^ by promoting the synthesis of new collagen. Furthermore, its ability to target melanin makes the 675 nm laser wavelength an effective and advantageous therapy for the treatment of melasma,^17^, ^18^, ^19^ even in darker phototypes.^20^

The clinical effectiveness of the 675‐nm laser in face rejuvenation was validated by a prospective observational study that involved 22 female participants who suffered from facial wrinkles. In all the cases, there was a reduction in wrinkles as measured by the Modified Fitzpatrick Wrinkles Scale assessment conducted both before and after three treatment sessions.^17^ Its efficacy in skin rejuvenation has also been successfully tested in the Asian phenotype as demonstrated by the recent investigation of Bonan et al.^21^

Additionally, Piccolo et al.^22^ findings supported the efficacy of the 675‐nm laser in minimizing wrinkles while improving skin texture, which can be attributed to the activation of dermal fibroblasts to generate new collagen. Furthermore, in younger patients who are genetically or chronically exposed to photoaging, the application of a 675‐nm laser system may be suggested due to its ability to increase collagen formation without having any adverse side effects,^7^ thus playing an important role in prejuvenation.^23^

In the field of trichology, it is known that red and near‐infrared lasers can prolong the anagen growth phase of the hair follicles (HFs), promoting an increase in hair count without significant side effects.^24^, ^25^ The laser technique may work by encouraging and prolonging the anagen phase of HFs, improving blood circulation, and stimulating fibroblasts to synthesize elastin and collagen. Collagen is an essential molecule in supporting the structure of HFs and promotes its healthy growth. Indeed, the administration of collagen peptides restores elasticity and strength, making the hair appear thicker and more full‐bodied by increasing the diameter of the hair shaft.^26^, ^27^

The mechanisms through which red light (620–700 nm) acts include photobiochemical reactions with an upregulation of intracellular oxidative stress and an increment of adenosine triphosphate (ATP) production. Reactive oxygen species (ROS) and transcription factors such as Nuclear Factor kappa B (NF‐kB) and hypoxia‐inducible factor‐1(HIF‐1) rise as a result of this cellular mechanism.^28^ Moreover, studies have reported that Insulin‐like Growth Factor 1(IGF‐1), Vascular Endothelial Growth Factor (VEGF), Fibroblast Growth Factor‐5 (FGF‐5), and FGF‐7 induce cell proliferation in the matrix, dermal papilla, and dermal papillary vascular system and increase the amount of extracellular matrix (ECM) in dermal papilla.^29^ These factors also maintain human hair follicles (HFs) in the anagen phase.^30^

The article "High‐powered 675‐nm laser: Safety and efficacy in clinical evaluation and in vitro evidence for different skin disorders" was retracted in 2026. Reasons: compromised peer review; unreliable results or conclusions; lack of ethics approval or compliance.

In addition to controlling protein synthesis, the transcription factors, as NF‐kB and HIF‐1, also affect tissue oxygenation, cytokines, growth factors, level of the inflammatory mediators, cell motility and proliferation. These processes play an important role in the formation of HFs promoting type 1 procollagen, metalloproteinase‐9 (MMP‐9), ECM production, and collagen synthesis through FGF activation, MMP‐1 reduction, angiogenesis stimulation, and blood flow enhancement.^31^

In this work, we first report the results of in vitro experiments obtained in cell cultures of human dermal fibroblasts subjected to irradiation with a 675 nm laser source, using various parameters related to the different fields of application. We then report the efficacy, the safety, the speed of treatment and post‐treatment outcomes in the management of skin rejuvenation/prejuvenation, acne scars, vascular lesions and pigmented lesions such as diffuse solar lentigines and melasma in which the high‐powered laser system emitting a 675‐nm laser system was applied.

## 2 MATERIALS AND METHODS

### 2.1 Device description

All patients were treated with Red Touch PRO laser system (DEKA M.E.L.A, Italy) which emits at a wavelength of 675 nm. Through the scanner, a fractional laser beam is emitted, and it is able to generate micro‐areas of selective thermal damage and denaturation (DOTs) of approximately 700 µm while leaving the epidermis unaffected by the integrated cooling system. A skin contact cooling handpiece (5°C) is included in the device to protect the epidermis from damage caused by the temperature rise. In addition, the scanner can be equipped with a contact sensor to increase patient safety. The study device can emit a maximum power of 15 W (50% more than the old setup).^14^ The handpiece is moved when the scanner has completed the entire scanning area. The laser allows the selection of several parameters including power, dwell time, spacing and stack. Specifically, the dwell time is the time the laser beam remains at the same point, while the stack indicates the number of laser pulses delivered consecutively at the same point. The power, dwell time and stack are used to change the energy that is emitted per single DOT (energy/DOT). In addition, the distance between the DOTs can be changed by the spacing value (Table 1).

The article "High‐powered 675‐nm laser: Safety and efficacy in clinical evaluation and in vitro evidence for different skin disorders" was retracted in 2026. Reasons: compromised peer review; unreliable results or conclusions; lack of ethics approval or compliance.

**TABLE 1:** The 675 nm laser parameters for each skin disorders.

Skin disease	Power	Dwell time	Spacing	Stack	Cooling	Energy/DOT	No. of treatments	Time interval between treatments	Follow‐up
***Pigmented lesions***:									
Diffuse solar lentigines	12–15 W	150 ms	1500 μm	1–3	5°C	1.8–6.75 J	1–3	30–45 days	6 months
Melasma	15 W	150 ms	1500 μm	1	5°C	2.25 J	1–3	30–45 days	6 months
***Skin rejuvenation***:									
Rejuvenation	15 W	150 ms	1500 μm	1–2	5°C	2.25–4.5 J	1–4	30–45 days	6 months
Prejuvenation	15 W	150 ms	1500 μm	1	5°C	2.25 J	1–2	30–45 days	6 months
**Acne scars**:									
Acne scars	15 W	150 ms	1500 μm	1–5	5°C	2.25–11.25 J	2–3	30–45 days	3 months
**Other treatments**:									
Acne vulgaris	15 W	150 ms	1500 μm	1	5°C	2.25 J	2	14–21 days	3 months
Vascular lesions	15 W	150 ms	1500 μm	1	5°C	2.25 J	10‐2	30–45 days	6 months

### 2.2 in vitro experiments on human cultured fibroblasts

Adult human dermal fibroblasts (hDFA) cells were purchased from Gibco, Life Technologies (Carlsbad, CA) and were used according to the manufacturer's instructions. Briefly, cells were cultured in a cell incubator (ICO50, Memmert GmbH, Germany), keeping the standard culture conditions (37°C and 5% CO_2_). The used culture medium is Dulbecco's Modified Eagle Medium (DMEM) low glucose, added with L‐Glutamine and Penicillin/Streptomycin, both 1% and foetal bovine serum (FBS) at 10%. Each reagent was purchased from PAN‐Biotech GmbH (Germany). In the experiments 2 × 10^4^ cells were cultivated in 35 mm imaging dish (µ‐dish 35 mm, low, Ibidi GmbH, Germany) and irradiated using 675‐nm laser device applying 390, 520 and 3.3 J/cm^2^ (parameter refers to the treatment of androgenetic alopecia (AGA)). One sample was left untreated and considered as a control. Irradiation was delivered working in a laminar flow biological hood, to maintain sterility in DMEM free of phenol red and FBS. Immediately after irradiation the samples were placed in incubators for 24 and 48 h.

### 2.3 Immunocytochemistry

At the appropriate time, the samples were fixed in paraformaldehyde solution (4% in saline phosphate buffer, PBS, PAN‐Biotech GmbH, Germany) for 6 min at room temperature (T_room_, 25°C). Two PBS washings were carried out for removing the fixative in excess and the immunocytochemistry protocol was applied. Cells were permeabilized in PBST solution containing 0.25% Triton X‐100 in PBS (Merck Life Science S.r.l., Milano, Italy) for 10 min at T_room_. The blocking of the nonspecific antibody binding was performed incubating hDFA cells for 30 min in PBS solution with 10% goat serum (PBSTG, Merck Life Science S.r.l., Milano, Italy). Cells were then incubated overnight at 4°C in primary antibody solution (PBSTG containing primary rabbit anti‐Ki‐67 antibody); the day after, hDFA cells were washed twice in PBS and incubated 1 h at T_room_ with AlexaFluor555‐labeled anti‐rabbit. Coverslips (18 mm) were mounted using Fluoroshield DAPI (Merck Life Science S.r.l) to stain cell nuclei. Each antibody was purchased from AbCam (Cambridge, UK) and used according with the manufacturing instructions. Ten immunocytochemical images were acquired for each sample using a SP8 laser scanning confocal microscope (Leica Microsystems, Mannheim, Germany), equipped with a  20X dry objective. The collected images were then analysed using the open‐source software (ImageJ, version 1.49v, National Institutes of Health, Bethesda, MD, USA).^32^

The article "High‐powered 675‐nm laser: Safety and efficacy in clinical evaluation and in vitro evidence for different skin disorders" was retracted in 2026. Reasons: compromised peer review; unreliable results or conclusions; lack of ethics approval or compliance.

### 2.4 Patient population and study design

Patients with pigmented lesions, superficial and deep wrinkles, fine line, acne scars were selected for this study. Exclusion criteria are: (i) hypersensitivity to light in the near‐infrared wavelength region, (ii) drug therapy based on anticoagulant and/or immunosuppressant and all types of active substances known to be photounstable or modifying their reactions as a result of sun exposure, (iii) pregnancy and breastfeeding, (iv) personal or family history of skin cancer, (v) patients who have been exposed to the sun in the 3 weeks before treatment, and (vi) patients suffering from light‐triggered seizure disorders.

Before the treatment, treated areas were cleaned and skin test was performed to determine the correct laser parameters. Minimum parameters were set according to the patient's phototype and lesion, and a small part of the area to be treated was irradiated. A thin layer of not coloured aqueous and transparent gel between the skin and the sapphire was placed. After 48–72 h, if the skin redness was minimal or absent, the parameters had to be increased, and if the redness was medium, the entire treatment area could be treated.

Patients were treated with one or more session with the study device depending on the severity of the skin disease (see Table 1).

After treatments, a moisturising emulsion to the skin was applied. In addition, the patient was asked to apply sunscreen and not to expose to the sun during the laser sessions and 3 weeks following the end of the treatment.

The article "High‐powered 675‐nm laser: Safety and efficacy in clinical evaluation and in vitro evidence for different skin disorders" was retracted in 2026. Reasons: compromised peer review; unreliable results or conclusions; lack of ethics approval or compliance.

### 2.5 Outcomes assessment

Serial clinical 3D Photos (3D LifeViz infinity, QuantifiCare, Biot, France) were collected before starting the treatment and during the follow‐up.

Depending on the treated skin disease, different assessment and validate scales for efficacy were used. The improvement of the skin was evaluated by using the 5‐point global aesthetic improvement scale (GAIS), where the observer gives a score from 0 to 4: 0 point, no change; 1 point, 25% mild improvement; 2 points, 50% moderate improvement; 3 points, 75% good improvement; 4 points, 100% excellent improvement. The patient satisfaction was measured using 5‐point (0–4) scale where 0 points indicated a very unsatisfied patient, 1 point indicated an unsatisfied patient, 2 point a neutral patient, 3 points a satisfied patient and 4 points a very satisfied patient. For the evaluation of rejuvenation treatments, the Fitzpatrick classification of wrinkling and degree of elastosis (FWCS Scale) was assessed at baseline and at follow‐up, a 9‐point scale where 1 point indicates fine textural changes with subtly accentuated skin lines and 9 points indicate multipapular and confluent elastosis approaching or consistent with cutis rhomboidalis.^33^

Finally, to assess patient safety, both side effects and patient‐perceived pain were monitored using a 5‐point scale: 0, no pain; 1, mild pain; 2, moderate pain; 3, severe pain; 4, intolerable pain.

### 2.6 Statistical analyses

In vitro data were reported as raw data, analysed used one‐way ANOVA followed post‐hoc test. Statistical significance was set at *p *< 0.05. All data were analysed using commercial software package GraphPad Prism 8th edition (GraphPad Software, San Diego, CA, USA).

Clinical data obtained from different scales were analysed using student's *t*‐test (one‐tail, paired). Statistical significance was set at *p *< 0.05. All outcome data were reported as means ± standard deviations (SD).

## 3 RESULTS

### 3.1 in vitro results

Irradiation of HDFa cells with the 675‐nm device did not induce Ki‐67 positivity after 24 h of irradiation (Figure 1A). After 48 h of treatment, the application of the fluence 390 J/cm^2^ induces a significant increase in Ki‐67^+^ cells (Figure 1B). Finally, after 72 h, both the application of 390 J/cm^2^ and the dose of 520 J/cm^2^ induce a significant increase in Ki‐67^+^ cells (Figures 1C and 2).

**FIGURE 1:** Ki‐67+ cell count irradiated with 675‐nm laser device applying fluences 390 and 520 J/cm^2^ (green and red column bars, respectively) after 24 (A), 48 (B) and 72 (C) h. The black column bar represents the control sample (non‐irradiated cells). Data were analysed by Kruskal–Wallis test followed Dunn's multiple comparisons test. Data were expressed as mean ± SEM (standard error of the mean), *N* = 2, *n* = 10. Statistical analyses: *p < 0.05; ***p < 0.001.

The article "High‐powered 675‐nm laser: Safety and efficacy in clinical evaluation and in vitro evidence for different skin disorders" was retracted in 2026. Reasons: compromised peer review; unreliable results or conclusions; lack of ethics approval or compliance.

**FIGURE 2:** Representative images obtained by confocal microscopy of (A) control samples (not treated) and (B) samples treated with 675‐nm laser. The nuclei of all HDFa cells are identified with DAPI, Ki‐67+ cells show colocalization of both markers. Scalebar: 100 µm.

Also, for androgenetic alopecia, additional preliminary in vitro experiments on hDFA cells were performed in order to test the effect of 675 nm laser on Ki‐67^+^ expression, demonstrating that the dose of 3.3 J/cm^2^ was able to stimulate cell proliferation already after 48 h following the laser treatment (Figure 3).

**FIGURE 3:** DAPI^+^ (A) cells and Ki‐67^+^ cells (B) in treated (grey column, 3.3 J/cm^2^ applied) and untreated samples (CTRL, black column, 0 J/cm^2^ applied). Data were analysed by Mann–Whitney two‐tailed test. Data were expressed as mean ± SEM (standard error of the mean), *N* = 2; *n* = 20. Statistical analyses: ***p < 0.001.

### 3.2 Clinical data

Skin rejuvenation/diseases treatments with 675 nm laser device were performed with different laser parameters according to treatment and patient's phototypes (Table 1). According to exclusion criteria, 11 patients with pigmented lesions, five patients with acne scars and 23 patients for rejuvenation treatments were included.

### 3.3 Pigmented lesions

#### 3.3.1 Diffuse solar lentigines

Eleven subjects with pigmented lesions were enrolled in the study. Six out of these patients showed diffuse solar lentigines on the face and décolleté area. Five patients were female and one was male: the age range was 38–55 years (average age 45.67 ± 6.19 years); the Fitzpatrick's index was II in two subjects and III in the remaining. Patients were treated with the following parameters: power 12–15 W, dwell time 150 ms, spacing 1500 µm, stack 1–3, cooling 5°C for an energy/DOT in the range of 1.80–6.75 J.

Immediately after treatment, all patients reached the paradoxical darkening leading to disappearance or the reduction of the number lesions at follow‐up (Figure 4).

**FIGURE 4:** Diffuse solar lentigines treatment with a 675 nm laser on a female patient's décolleté. The baseline (A) and the follow‐up after 6 months from the last treatment (B) are shown.

The mean GAIS score was 3.67 ± 0.52 points and patient satisfaction was 2.83 ± 0.41. Regarding safety, only 1 patient showed temporary slight redness and all the six subjects showed mild crusts which disappeared in 7–10 days. The average pain score obtained was 1.50 ± 0.55.

The article "High‐powered 675‐nm laser: Safety and efficacy in clinical evaluation and in vitro evidence for different skin disorders" was retracted in 2026. Reasons: compromised peer review; unreliable results or conclusions; lack of ethics approval or compliance.

#### 3.3.2 Melasma

The five remaining patients (five females, Fitzpatrick skin type III, mean age 38.6 ± 9.07) showed melasma on their face that were irradiated with 675‐nm using the following parameters: power 15 W, dwell time 150 ms, spacing 1500 µm, stack 1, cooling 5°C for an energy/DOT of 2.25 J.

Even in previous cases, a reduction or complete resolution of the characteristic hyperpigmentation of melasma was observed. The scores obtained in the different features studied are indicated as follows: GAIS: 3.20 ± 0.45; patient satisfaction: 3.00 ± 0.00; pain: 1.40 ± 0.55. Immediately after treatment, one patient showed erythema that resolved in 24 h and four patients showed mild‐moderate crusts that disappeared in 3–7 days. No severe adverse effects were reported.

#### 3.3.3 Skin rejuvenation

Sixteen patients (15 females and one male), of which seven patients with Fitzpatrick skin type II and nine with Fitzpatrick skin type III, with a mean age of 50.88 ± 5.73 years, underwent 1–4 facial rejuvenation treatments. The laser treatment was applied with the following parameters: power 15 W, dwell time 150 ms, spacing 1500 µm, stack 1–2, cooling 5°C and an energy/DOT between 2.25 and 4.5 J.

During the follow‐up visit, patients showed improvement in texture, pores, skin laxity, increased volume and decreased wrinkles (Figure 5). These improvements were also assessed quantitatively by FWCS score (2.92 ± 2.47 points at baseline and 2.00 ± 1.48 points at follow‐up; *p *< 0.05), GAIS score (2.93 ± 0.88) and patient satisfaction scale (2.44 ± 0.73). Pain was assessed with a mean score of 1.20 ± 0.41. All patients showed diffuse redness immediately after treatment (typical endpoint for skin rejuvenation treatments), which resolved within a few hours, but for four patients it lasted for about 1–2 days. Thirteen out of 16 patients reported light crusts that disappeared in 2–7 days.

**FIGURE 5:** Full face laser skin rejuvenation treatment in female patient at baseline (A) and at 6 months follow‐up after the last treatment session (B). Smoothed wrinkles are observable in the perioral area at 6 months follow‐up after the last treatment.

#### 3.3.4 Prejuvenation

Seven women with an average age of 38.43 ± 6.48 years (six patients with phototype III and one with phototype II) underwent one or two treatments with the following parameters: power of 15 W, dwell time 150 ms, spacing 1500 µs, stack 1, cooling 5°C and energy/DOT of 2.25 J. As in the previous case, the patients showed good results (Figure 6) as measured by GAIS score (3.40 ± 0.89) and satisfaction (2.83 ± 0.41). The FWCS score did not present statistically significant results. Regarding side effects, one patient showed slight redness for 1 day, while 50% of patients reported mild crusting that resolved in 2–3 days. Pain score was 1.00 ± 0.00.

The article "High‐powered 675‐nm laser: Safety and efficacy in clinical evaluation and in vitro evidence for different skin disorders" was retracted in 2026. Reasons: compromised peer review; unreliable results or conclusions; lack of ethics approval or compliance.

**FIGURE 6:** Full face laser skin prejuvenation treatment in female patient at baseline (A) and at 6 months follow‐up after the last treatment session. A visible improvement in the perioral and periocular area at 6 months follow‐up after the last treatment was observed.

#### 3.3.5 Acne scars

Five patients with acne scars (three females and two males, average age 36.00 ± 9.54, three subjects with skin type II, and two with skin type III) were treated with 2–3 sessions of 675‐nm laser with the following parameters: power 15 W, 150 ms, 1500 µm, stack 1–5 for an energy/DOT between 2.25 and 11.25 J.

The acne scars flattened, the skin regained some of the lost volume and the patient had an overall improvement in texture (Figure 7).

**FIGURE 7:** The 675 nm laser treatment of acne scars in cheek area of female patient. The baseline (A) and the follow‐up after 3 months from the last treatment (B) are shown.

Patients were assessed by GAIS score (3.50 ± 0.58) and their satisfaction after treatment (2.75 ± 0.50). Pain was assessed with 1.00 ± 0.00 point, so patients found this treatment mild painful. As in previous patients, if redness and crusts were reported, they disappeared in a maximum of 7 days.

#### 3.3.6 Other treatments

Some patients included in the study for the treatment of skin rejuvenation, melasma or diffuse pigmented lesions treatments showed improvements in other skin diseases such as acne vulgaris and diffuse vascular lesions.

#### 3.3.7 Acne vulgaris

Two patients (two females, average age 31.50 ± 9.19 years, Fitzpatrick skin type III) with acne vulgaris were treated with two laser sessions: power 15 W, dwell time 150 ms, spacing 1500 µm, stack 1 for an energy/DOT of 2.25 J. At the follow‐up visit, the patients showed a reduction in the number of acne lesions and an improvement in skin texture (Figure 8).

**FIGURE 8:** Female patient treated with 675 nm laser at baseline (A) and at 3 months follow‐up months from the last treatment session (B). The photos show a reduction in the number of acne lesions in the cheek area.

The Global Score scale showed an average score of 3.5 ± 0.71 and both patients were satisfied with their results (3.00 ± 0.00). The pain score was also reconfirmed in these clinical cases (1.00 ± 0.00).

#### 3.3.8 Vascular lesions

One patient with rosacea and two patients with diffuse redness (two females and one male, average age 49.00 ± 5.57 years, Fitzpatrick skin type II‐III) were treated: power 15 W, dwell time 150 ms, spacing 1500 µm, stack 1, cooling 5°C and an energy/DOT of 2.25 J.

The article "High‐powered 675‐nm laser: Safety and efficacy in clinical evaluation and in vitro evidence for different skin disorders" was retracted in 2026. Reasons: compromised peer review; unreliable results or conclusions; lack of ethics approval or compliance.

The irradiated skin showed improved brightness and texture and a significant reduction of the vascular component in the full face (Figure 9).

**FIGURE 9:** Female patient treated with 675 nm laser at baseline (A) and at 6 months of follow‐up from the last treatment session (B). Photos of the same patient acquired with the filter for the vascular component before (C) and at 6 months of follow‐up from the last treatment session (D).

The GAIS scale and the patient satisfaction scale reported were 3.33 ± 0.58 and 3.00 ± 0.00, respectively. The average pain value was 1.67 ± 0.58 and only few patients reported mild redness for the first 2 days and mild crusting for another 2–3 days.

## 4 DISCUSSION

The treatment of skin disorders such as acne scars, pigmented or vascular lesions and deep/fine wrinkles remains a challenge in aesthetic medicine. Even though there are several techniques for improving the appearance of skin, it is crucial to find additional, tolerable options for minimizing patient's^34^ downtime. Different therapies are available to manage skin disorders, among them the use of ablative and non‐ablative lasers. The potential risks associated with non‐ablative lasers are far less than those associated with ablative lasers.^35^

Fibroblasts are one of the major cellular components present in the dermis. Among their main functions are the synthesis of collagen, both in physiological conditions for the maintenance of tissue homeostasis, but also during the wound healing process. They also contribute to continuous ECM remodeling.^36^ During ageing, the number of dermal fibroblasts is reduced physiologically. This leads to loss of elasticity by the skin and formation of wrinkles, as well as other effects related to aging.^37^, ^38^ As observed with previous experiments conducted in HDFa cells with different methods.^7^ in vitro tests on cultured human fibroblasts showed that the application of 390 and 520 J/cm^2^ emitted with a source at 675 nm does not induce cytotoxic effects.

Here, we used a known marker in order to detect cell proliferation, named Ki‐67. This protein is highly conserved, and its expression is observed in all phases of the cell cycle, except for G_0_ and in quiescent cells. It is found as a constituent of heterochromatin in the early stages of the G_1_ phase and in the nucleolus in the late G_2_ phase of the cell cycle. In addition, the decrease in its mRNA levels is correlated with a reduction in the rate of cell proliferation.^36^ Recent studies showed that suppression of Ki‐67 expression in several non‐tumorigenic cell lines results in increased expression of the cyclin‐dependent kinase inhibitor 1 (CDK inhibitor p21), which leads to a reduction in the S‐phase cell portion. Despite this, the amount of DNA did not vary and cell proliferation was not compromised.^13^ The Ki‐67 was also used in in vivo experiments to study the healing process after a single helium‐neon laser exposure. In particular, the formation of granulation tissue and the presence of Ki‐67^+^ cells in the basal layer of the epidermis were observed after 10 days.^39^

The article "High‐powered 675‐nm laser: Safety and efficacy in clinical evaluation and in vitro evidence for different skin disorders" was retracted in 2026. Reasons: compromised peer review; unreliable results or conclusions; lack of ethics approval or compliance.

Our results obtained by quantifying HDFa cells positive to Ki‐67, show that the dose of 390 J/cm^2^ stimulate cell proliferation already after 48 h after treatment, while the dose of 520 J/cm^2^ stimulates it after 72 h. Even a minimum dose of 3.3 J/cm^2^ stimulates Ki‐67 expression for up to 48 h after treatment. At the same time the nuclear morphology observed by staining with DAPI does not suggest cytotoxic effects or induction of apoptosis. These results suggest that the application of the wavelength at 675‐nm can stimulate fibroblasts proliferation. Furthermore, already published data on cultured HFs have demonstrated that red light enhances Ki‐67 positive cells.^40^

Indeed, the existing literature, Zheng et al.^41^ demonstrated that the increase of collagen production creates a more favourable microenvironment for HFs. These advantageous conditions expedite the transition of HFs into the anagen phase, consequently promoting hair growth. The mechanism of action by which collagen peptides promote hair regeneration is linked to their ability to reduce tumour necrosis factor‐alpha (TNF‐α) and interleukin‐1beta (IL‐1β) in HFs, hence aiding in the regulation of inflammatory reactions that may arise in individuals with AGA.

From the point of view of clinical use, the 675‐nm laser device does not induce hyperpigmentation and it can be used on patients with darker phototype.^42^ Non‐ablative lasers, such as the 675‐nm technology, promote neocollagenesis by dermal fibroblasts.^7^ Furthermore, 675 nm laser has also proven to be effective in the treatment of androgenetic alopecia,^43^ and dorsal hand skin hyperpigmentation.^44^

There are many potential explanations for the increased number of HFs. First, angiogenesis is linked to active hair growth,^45^ and VEGF, a crucial angiogenesis component, has been shown to operate as a mediator of HFFIVEs growth and cycling. Furthermore, the increase of collagen production creates a more favourable microenvironment for HFs.^41^ From our investigation the results obtained after the irradiation with the dose of 3.3 J/cm^2^ of hDFA cultures showed an increase of Ki‐67^+^ expression, demonstrating that this low dose is able to stimulate cell proliferation already after 48 h following the laser treatment. The 675 nm wavelength directly affects the component of collagen in skin and it is minimal absorbed by the vascular constituent of the dermis, representing a potential therapeutic option for acne scarring and other skin conditions. Consequently, there was a lower risk of adverse effects and post‐treatment patient's maintenance.

The article "High‐powered 675‐nm laser: Safety and efficacy in clinical evaluation and in vitro evidence for different skin disorders" was retracted in 2026. Reasons: compromised peer review; unreliable results or conclusions; lack of ethics approval or compliance.

The mechanism of action is represented by the production of a thermal column that transfers heat to the surrounding tissues, causing rapid denaturation and shrinkage of collagen in addition to the formation of new collagen and the resulting ‘softening’ of scars and general improvement in skin texture.^42^

The technique utilized in this study offers a wide range of possible combinations of the operating parameters to address the symptoms of different skin conditions. Particularly the great advantage of this new technology compared with the old one, in which a power value of 10 W was selected,^14^, ^15^, ^16^, ^17^, ^20^, ^21^, ^22^, ^42^ is represented by the use of a higher level of power (15 W instead of 10 W) which allows the operator to perform a faster treatment session (reducing the treatment time) while using the same level of energy.

In order to demonstrate the safety and effectiveness of the high‐power 675‐nm laser system, the overall data were evaluated to give a single response and to assess possible differences in results depending on the treated skin disease.

With the use of validated scales like 5‐points GAIS and patient's satisfaction scale the findings of the current study showed that the high‐powered 675 nm laser led to promising and good results for all skin pathologies treated with a treatment time that was reduced by 50% compared to the old parameters setting, resulting in a faster and good patient's satisfying treatment technique.

Indeed, the Global score using 5‐point scales showed values between 3 and 4 points for all treated pathologies, all scores between ‘75%‐good improvements’ and ‘100%‐excellent improvements’ (Figure 10). Concerning pigmented and vascular symptoms, the average GAIS values found in this study appeared to be greater than those measured in previously published studies such as that of Corricciati et al.,^18^ where the GAIS for visible, pigmentary and vascular values were, respectively, 1.89 ± 0.96, 2.28 ± 0.67 and 2.17 ± 0.79.

**FIGURE 10:** Graphical representation of mean values and standard deviation of GAIS scores for each skin disorder treated with 675 nm laser.

The assessment of patient satisfaction showed in Figure 11 confirms the previous data: all average values are between 2 and 3 points (between ‘satisfied’ and ‘very satisfied’) (maximum score allowed by this scale). Finally, the average pain values shown mild and moderate pain perceived (Figure 12). No statistically significant results were found for the FWCS score. Probably, this scale is not the appropriate tool for quantifying improvements in patients with very slight and superficial skin imperfections.

The article "High‐powered 675‐nm laser: Safety and efficacy in clinical evaluation and in vitro evidence for different skin disorders" was retracted in 2026. Reasons: compromised peer review; unreliable results or conclusions; lack of ethics approval or compliance.

**FIGURE 11:** Graphical representation of mean values and standard deviation of Patient's assessment scores for each skin disorder treated with 675 nm laser.

**FIGURE 12:** Graphical representation of mean values and standard deviation of perceived pain score for each skin disorder treated with 675 nm laser.

Concerning safety, all patients showed the same undesirable effects: a slight initial redness and the formation of mild crusts which disappeared within a maximum of 1 week.

Furthermore, this technique has shown to be effective as prejuvenation treatment, supporting to maintain and to preserve a youthful appearance starting from young ages.^23^ In this scenario, younger individuals who have been genetically or chronically exposed to photoaging may benefit from the use of a laser that can increase collagen formation without having any adverse reactions.^7^

## 5 CONCLUSION

The application of the high‐power 675 nm laser has proven effective in stimulating cell proliferation in in vitro experiments.

Furthermore, the high‐powered 675 nm laser has shown excellent results on various skin conditions including diffuse pigmented lesions, melasma, skin rejuvenation, acne scars, acne vulgaris and vascular lesions, and patients treated have reported no serious adverse effects. Furthermore, with this new technology, faster treatments can be carried out compared to the previous system. In conclusion, the clinical data confirm the efficacy and safety of this high‐powered 675 nm laser.

## CONFLICT OF INTEREST STATEMENT

Tiziano Zingoni, Laura Pieri, Francesca Madeddu and Irene Fusco were employed by El.En. Group. The remaining authors declare that the research was conducted in the absence of any commercial or financial relationships that could be construed as a potential conflict of interest.

## INSTITUTIONAL REVIEW BOARD STATEMENT

The article is in accordance with the Declaration of Helsinki on Ethical Principles for Medical Research involving human subjects. Ethical approval is not necessary as the study device is already CE marked since 2019.

## INFORMED CONSENT STATEMENT

Informed consent was obtained from all subjects involved in the study.

## Data Availability

Data available on request from the authors.
